# Network Intrusion Detection Method Combining CNN and BiLSTM in Cloud Computing Environment

**DOI:** 10.1155/2022/7272479

**Published:** 2022-04-28

**Authors:** Jing Gao

**Affiliations:** School of Information and Mechatronics Engineering, Zhengzhou Business University, Henan, Gongyi 451200, China

## Abstract

A network intrusion detection method combining CNN and BiLSTM network is proposed. First, the KDD CUP 99 data set is preprocessed by using data extraction algorithm. The data set is transformed into image data set by data cleaning, data extraction, and data mapping; Second, CNN is used to extract the parallel local features of attribute information, and BiLSTM is used to extract the features of long-distance-dependent information, so as to fully consider the influence between the front and back attribute information, and attention mechanism is introduced to improve the classification accuracy. Finally, C5.0 decision tree and CNN BiLSTM deep learning model are combined to skip the design feature selection and directly use deep learning model to learn the representational features of high-dimensional data. Experimental results show that, compared with the methods based on AE-AlexNet and SGM-CNN, the network intrusion detection effect of this method is better, the average accuracy can be improved to 95.50%, the false-positive rate can be reduced to 4.24%, and the false positive rate can be reduced to 6.66%. The proposed method can significantly improve the performance of network intrusion detection system.

## 1. Introduction

With the continuous development of technologies such as distributed computing, grid computing, and parallel computing, cloud computing has emerged [1]. The principle of cloud computing is to allocate computing tasks in a large-capacity resource pool. These resource pools are not remote servers or computer entities, but are composed of a large number of distributed computers. Enterprises and users access computers and storage systems according to their needs [2–4]. In the past experience, companies and users are more accustomed to obtaining data on local computers. The resource pool of cloud computing is not located on local computers but on distributed computers. Therefore, it has brought great changes to the user's operating habits [5]. In addition, the cost of use has been reduced, and the traditional “point-to-point” information dissemination method has been transformed into a multiperson sharing information dissemination method that greatly improve the efficiency and convenience of users to obtain information [6]. Cloud computing has the characteristics of high reliability, measurable service, virtuality, and low cost. These just solve the problems of the Internet big data era and also bring broad development opportunities for many enterprises and individuals [7].

Cloud computing can not only bring technical support to the development of enterprises, but also a cross-age symbol of information technology. On the other hand, although the development situation of cloud computing is very good, the obstacles behind it cannot be ignored. In particular, the issue of network security has become the most concerned issue. The huge commercial value of cloud computing is very attractive to intruders. According to the principle of cloud computing, the remote cloud handles the storage and reading of a series of data. It is also because of this that its service providers and users are vulnerable to various forms of attacks. Including man-in-the-middle attacks, network sniffing, denial of service attacks, port scanning and other attack forms [8–10]. Once the cloud is subjected to these cyber attacks, user data and privacy may be lost or leaked. If the target of the attack is a large enterprise or government department, it may cause social unrest and even threaten national security. In recent years, cloud security accidents have occurred frequently, and each time has caused serious economic losses to enterprises and society.

In 2007, cloud computing attracted widespread attention in the industry and made great progress at home and abroad. Because of the obvious advantages of cloud computing, the industry at that time put more attention on popularizing cloud computing and did not consider the security of cloud computing too much. The recent series of cloud security incidents are also telling people the importance of strengthening cloud computing security. International research on cloud security has just started. Although many organizations and institutions conduct analysis and research on cloud computing security issues, it is mainly the Cloud Computing Alliance (CSA) and Microsoft, Google, Amazon, and other organizations that have put forward a basic understanding of cloud computing security and preliminary solutions for cloud computing security. 

The intrusion detection system has a development history of more than 30 years, and it has gradually developed into a commercial market product. And it has become the main research topic and direction of Internet security [11–13]. The system model is composed of subjects, objects, audit records, profile features, abnormal records, and activity rules. In 1989, the US National Computer Security Center developed the host-based anomaly detection system W&S (Widsom and Sence). In 1990, the University of California at Davis developed the NSM intrusion detection system. The system is used to analyze the network data packets of the local area network and detect abnormal attack behaviors. It is not an analysis of data records in the host, but a network-oriented intrusion detection system. In 1992, the CMDS misuse detection system developed by SAIC was the first intrusion detection system to be applied to commercial purposes. In 2000, E. Spafford and D. Zamboni proposed an intrusion detection autonomous agent system. So that intrusion detection has the characteristics of being distributed and adaptive [14–16]. Intrusion detection technology is constantly evolving and updating. Technologies such as data mining, pattern recognition, rough sets, support vector machines, and neural networks have been continuously applied to intrusion detection systems [17]. Continuously improve and improve the efficiency of intrusion detection, pushing the development of intrusion detection to a new height [18].

Traditional intrusion detection models based on deep learning algorithms often use Softmax single classifiers for classification in the output layer. In the face of massive high-dimensional data, due to the impact of data dimensions, the training model often leads to a low detection rate of attacks, which affects the overall detection efficiency. The use of deep learning to build an intrusion detection system can extract higher-dimensional features from the original data, thereby obtaining a better classification model. In order to improve the accuracy of network intrusion detection, the main innovations of this paper are as follows:

1. Design a model that integrates CNN and BiLSTM networks. The parallel local features and long-distance dependent features of the information are extracted, and the attention mechanism is introduced to improve the classification accuracy of the model.
2. Combine C5.0 decision tree and CNN-BiLSTM deep learning model. Skip the design feature selection method and directly use the deep learning model to learn the characterization features of high-dimensional data, which further improves the detection accuracy of the algorithm.

## 2. Related Research

At present, the commonly used deep learning algorithms for network intrusion detection include DNN-based algorithms [19], BP neural network-based algorithms [20], convolutional neural network (CNN)-based algorithms, recurrent neural network (RNN)-based algorithms, and algorithms based on algorithm of deep belief network. Compared with traditional machine learning methods, deep learning methods have a greater improvement in detection performance, but there are still some shortcomings [21]. In terms of feature extraction, although CNN can learn local features in time or space and avoid the manual extraction process, it lacks the ability to learn sequence correlation. Therefore, the problem of long-term dependence on longer information cannot be solved. Long-short term memory (LSTM) feature extraction has a high accuracy rate and can solve the problem of long-term dependence, but its false alarm rate is relatively high. And because LSTM can only read sequence data in one direction, it cannot fully consider the impact of subsequent attribute information. In terms of feature learning, deep learning algorithms fail to explain the correlation between features and category labels. In terms of adaptability, how to make the model have the ability to adaptively update without reducing the accuracy rate and increasing the false alarm rate is still to be further studied. In addition, the attention mechanism [22, 23] algorithm is widely used in natural language processing, text classification, and other fields and can achieve good classification results. But it is rarely used in network intrusion detection. Gao et al. [24] introduced the deep belief network into the field of anomaly detection and composed a neural network classifier with a multilayer-restricted Boltzmann machine and use the deep belief network and support vector machine (SVM) model on the KDD99 data set for comparison. Tang et al. [25] applied deep learning methods to software-defined networking (SDN) environment for anomaly detection. And the experiment is carried out on the NSL-KDD data set. The results also show that deep learning methods have strong potential in stream-based anomaly detection in SDN environments. Javaid et al. [26] et al. carried out network intrusion detection based on self-taught learning (STL). This algorithm makes the detection system more flexible and efficient in detecting abnormal events. Vinayakumar et al. [27] used CNN for network intrusion detection, modeling network traffic as a time series. Similarly, the KDD99 data set proves the effectiveness of its network structure in intrusion detection. Alqat et al. [28] proposed an effective deep learning method based on the STL framework. It greatly reduces the detection time of the network intrusion detection system and effectively improves the accuracy of the support vector machine for attacks. Chen and Chen [29] merged ResNet and BiLSTM networks to build an IoT intrusion detection classification model. The optimization method has achieved good results in two aspects of classification accuracy and efficiency. Dong et al. [30] proposed a dimensionality reduction method for intrusion detection based on self-encoding, which preprocessed intrusion detection data. The model uses an automatic coding AlexNet neural network. Zhang et al. [31] designed a stream-based intrusion detection model SGM-CNN. Combine unbalanced processing with CNN. The UNSW-NB15 and CICIDS2017 data sets are used to verify the superiority of the proposed model. Wang [32] found that deep neural networks are vulnerable to adversarial examples in the field of image classification. That is, they provide some opportunities for attackers to misclassify the network by introducing unperceptible changes to the original pixels in the image.

## 3. Related Work

### 3.1. CNN-Based Network Intrusion Detection Method

In the field of network intrusion detection, CNN is a hierarchical model, which has good performance in extracting local features. A typical CNN model usually combines the three ideas of local receptive fields, shared weights, and spatial or temporal sampling. This gives it a unique advantage when dealing with data with statistical stability and local relevance. The principle block diagram of the network intrusion detection system based on CNN is shown in Figure 1.

The workflow of a CNN-based network intrusion detection system can be divided into 4 steps:

Step 1: Preprocess each record in the intrusion detection data set so that its data type format can be used as the input of the CNN model.
Step 2: The processed data are input to the input layer of CNN, and then the convolution layer performs convolution operation on it to accurately extract the characteristic information of each record.
Step 3: The pooling layer integrates the feature points in the small neighborhood to obtain new features. The purpose of pooling operation is to speed up network training. Commonly used methods are average pooling and maximum pooling.
Step 4: Data are input into the Softmax classifier through the fully connected layer to classify the intrusion type.

CNN-based network intrusion detection methods are superior to traditional methods in classification accuracy and can accurately extract local feature information. However, this method is still lacking in learning sequence correlation information and cannot solve the problem of long-term dependence. Its accuracy rate needs to be improved.

### 3.2. LSTM-Based Network Intrusion Detection Method

RNN is good at processing sequence data. However, in the training process, there will be problems of gradient disappearance, gradient explosion, and long-term dependence. The long- and short-term memory module in the LSTM model can solve the long-term dependence problem caused by RNN. The LSTM module adds 3 gates and a cell state update to the hidden layer of the RNN model, as shown in Figure 2.

The forget gate screens the state of the upper layer of cells, leaving useful information and forgetting useless information. The calculation formula is as follows:

(1) $$\begin{array}{c} f_{j}=\delta \left(b_{f}+w_{f}\cdot \left[h_{j-1},x_{j}\right]\right), \end{array}$$

where **w**_*f*_ and **b**_*f*_ are the weight matrix and the bias term of the forget gate, respectively, **h**_*j*−1_ is the output value of the upper LSTM, *δ* is the sigmoid activation function, and [,] means to connect two vectors into one vector.

The input gate judges the importance of the information and sends the important information to the cell state update place to complete the update of the cell state. The process consists of 2 parts. The first part uses the sigmoid function to determine the new information that needs to be added to the cell state. Part 2 applies the tanh function to generate a new candidate vector. The calculation process is

(2) $$\begin{array}{c} \left\{\begin{array}{c} f_{j}=\delta \left(b_{i}+w_{i}\cdot \left[h_{j-1},x_{j}\right]\right),\\ c_{j}=\tanh\left(b_{c}+w_{c}\left[h_{j-1},x_{j}\right]\right), \end{array}\right. \end{array}$$

where **w**_*i*_ and **b**_*i*_ are the weight and bias of the input gateand **w**_*c*_ and **b**_*c*_ are the weight and bias of the cell state. After the above processing, the original cell state **c**_*j*−1_ is updated to the current cell state **c**_*j*_. The update formula is

(3) $$\begin{array}{c} c_{j}=i_{j}*{\tilde{c}}_{j}+f_{j}*c_{j-1}, \end{array}$$

where ∗ represents the element multiplication operation, **f**_*j*_^*∗*^**c**_*j*−1_ means to delete information, and $i_{j}*{\tilde{c}}_{j}$ represents newly added information.

The output gate controls the output of the cell states of this layer and determines which cell states are input to the next layer. The calculation formula is

(4) $$\begin{array}{c} \left\{\begin{array}{c} o_{j}=\delta \left(b_{o}+w_{o}\cdot \left[h_{j-1},x_{j}\right]\right),\\ h_{j}=o_{t}*\left.\tanh\left[c_{j}\right]\right). \end{array}\right. \end{array}$$

The network intrusion detection method based on LSTM first digitizes, standardizes, and normalizes the original detection data set. Then input the preprocessed data set into the trained LSTM model. Finally, the result of the LSTM model is input into the classifier to obtain the classification result. This method can extract more comprehensive features and improve the accuracy of network intrusion detection when processing sequence data, but its false alarm rate is relatively high.

### 3.3. C5.0 Decision Tree Classification Model

The C5.0 decision tree classification algorithm is a new classification algorithm based on the C4.5 classification algorithm. The decision tree construction idea of C5.0 algorithm is consistent with that of C4.5 algorithm. The C5.0 algorithm also includes all the functions of the C4.5 algorithm. The difference from the C4.5 algorithm is that the C5.0 algorithm introduces boosting technology and cost matrix construction technology.  Figure 3 is a schematic diagram of boosting integration. The application of boosting technology to C5.0 classifier is one of the important improvements of C4.5 algorithm. The algorithm trains the samples to adjust the weight value. By learning multiple classifiers, these classifiers are combined linearly to achieve the purpose of improving the classification accuracy.

## 4. Proposed Model

### 4.1. Detection Model

This paper first performs data cleaning, data extraction, and data mapping preprocessing on the KDDCUP99 detection data set. Use CNN to extract local parallel features to obtain more comprehensive local features. In order to solve the influence of the front and back features of each attribute feature point on the attribute feature point, a BiLSTM model composed of 4 memory modules is used to extract long-distance dependent features. Each module consists of a topological structure of 2 cells. Finally, the attention mechanism is used to calculate the importance of each attribute feature. The classification result is obtained through the C5.0 classifier to improve the accuracy rate and reduce the false alarm rate. The principle block diagram of the algorithm in this paper is shown in Figure 4.

### 4.2. Data Preprocessing

In order to build an IoT intrusion detection classification model based on the fusion of CNN and BiLSTM, it is necessary to preprocess the original data set using steps such as data cleaning and data transformation.

“Dirty data” refers to incomplete, noisy, and inconsistent data. The internal laws in the original data information are destroyed, resulting in poor performance of data analysis and processing. Therefore, it is necessary to clean the “dirty data” and convert the “dirty data” into data that meets the data quality requirements. The main problems faced by data cleaning are missing values, erroneous data, outliers and noise. The solution is to use the same constant to fill in the missing data set and to clear or replace the existing special symbols and garbled codes.

In this paper, the KDD CUP 99 test data set includes 34-bit numerical attributes and 7-bit character attributes. In order to increase the difference between samples of different categories and improve the classification effect of the model, this paper proposes a data extraction algorithm to preprocess the original data set. Suppose the sample space *T*={*T*_1_, *T*_2_,…, *T*_*n*_}, the current sample is *T*_*t*_, and the sample category *i*={0,1,2,3} represents denial of service attacks, unauthorized remote access, scanning and probing, and illegal access to local users. The pseudo code of the data extraction algorithm is shown in Algorithm 1.

After the above operations, continue to map the data in the data set *D*_*B*_ to the image data set. In this paper, the window size is set to *w* = 10, and the number of features in the KDD CUP99 detection data set is 42. Therefore, the matrix *W* with a size of 10 × 42 in the data set *D*_*B*_ is mapped to a grayscale image with a size of 10 × 42. Each pixel in the image corresponds to the value of the corresponding position in the matrix. However, since the value range of the gray scale image is [0, 255], the data interval in the original matrix *W* is relatively large. In order to retain more feature details, the original matrix *W* needs to be normalized during the mapping. At present, the commonly used normalization methods include mean variance normalization and maximum minimum normalization. The data after the normalization of the mean variance conform to the standard normal distribution. It is commonly used in some clustering algorithms that obtain similarity through distance. The calculation formula is

(5) $$\begin{array}{c} x=\frac{x-\bar{x}}{\partial }, \end{array}$$

where *x* is the current value of a certain data in the sequence; $\bar{x}$ is the mean value of the data in the series; and ∂ is the standard deviation of the sequence.

### 4.3. CNN-BiLSTM Network Feature Extraction

Both CNN and BiLSTM are classic models in deep learning. The CNN network can use the hidden layer to learn the local features of the data layer by layer and extract the data features in the spatial dimension. BiLSTM network has the characteristics of long-term preservation of contextual historical information and can extract features in the time dimension. Therefore, this section uses CNN and BiLSTM to build a CNN-BiLSTM neural network model to learn the temporal and spatial characteristics of the data set.

The main parameters of the CNN-BiLSTM neural network module are in the CNN-BiLSTM network, the activation function is set to Relu, the optimization function is Rmsprop, and the learning rate is 0.0001. In addition, the loss function loss used by different numerical methods is also different. The numerical method in this paper is not one-hot, but directly uses numerical coding. So use Sparse Categori-Calcrossentropy as the loss function.

Figure 5 shows the number of layers of the CNN-BiLSTM neural network model and the parameters of each layer. In the CNN-BiLSTM model, the samples are first input into the CNN, and four one-dimensional convolution operations and two sampling operations are performed. The tensor of the input sample is (None, 41, 64), where None is a placeholder for the size of the input sample. After the CNN operation, the obtained (None, 10, 128) tensor is input into the BiLSTM network. The first dense layer is the middle layer for extracting features, and the number of output features is controlled by changing the number of nodes. Finally, the (None, (5∼40)) tensor output by the last fully connected the dense layer.

In the process of training the model, the optimal model parameters are found by adjusting the epoch value, the learning rate, and the number of nodes in the dense layer.  Figure 6 shows the acc-loss change curve of the algorithm on the KDD CUP 99 data set. When the epoch value is between 120 and 160, the Dese value is 25, and the learning rate is 0.0001, the training acc value on the KDD CUP 99 data set is 99.73%, and the training loss value is 0.51%. At this time, the performance of the CNN-BiLST model has reached a good level.

### 4.4. Attention Mechanism Layer

In order to improve the classification accuracy, the result of CNN-BiLSTM is input to the attention mechanism layer. The treatment process is shown in formulas (6)–(8).

(6) $$\begin{array}{c} u_{t}=\tanh\left(W_{w}P_{t}+b_{w}\right), \end{array}$$

(7) $$\begin{array}{c} a_{t}=\text{softmax}\left(u_{t}^{T},u_{w}\right), \end{array}$$

(8) $$\begin{array}{c} v=\sum a_{t}P_{t}, \end{array}$$

where **u**_*t*_ is the attribute representation of **P**_*t*_, **W**_*w*_ is the context vector, which is randomly generated during the training process, **a**_*t*_ is the importance weight, and **v** represents the high-level representation obtained by performing importance weighted summation on **P**_*t*_.

Finally, input the output result **v** of the attention mechanism layer into the C5.0 classifier to obtain the classification result.

The CNN-BiLSTM model has the following characteristics:

1. The one-hot preprocessing method is used to convert symbolic features into numerical features. Compared with other pretreatment methods, the conversion efficiency can be improved.
2. Using the advantages of the CNN model for local parallel feature extraction, the attribute feature extraction operation is performed to solve the problem of local feature loss.
3. Based on the advantages of LSTM in processing long sequence data, the BiLSTM model is used to extract long-distance-dependent features. Consider the influence of the attributes before and after each attribute point in the sequence data on the feature extraction, so as to achieve the purpose of reducing the false alarm rate of network intrusion detection.
4. The attention mechanism is introduced to calculate the importance of each attribute feature. Pay more attention to important features to get a better intrusion detection effect.

### 4.5. C5.0 Classifier Training

In the proposed model, the boosting algorithm is added to the C5.0 algorithm through the C5.0 function. In the C5.0 function, the role of the trials parameter is to control the number of C4.5 decision trees and to enhance the classification performance of the C5.0 model. After constructing the C5.0 classifier, start training the C5.0 classifier. By adjusting the specific values of parameters such as trials, the model is optimized, so that the model can achieve better classification performance.

## 5. Validation of Calculation Examples and Discussion of Results

### 5.1. Experimental Environment and Data Set

In order to verify the effectiveness of the model checking algorithm, this paper uses Windows 10 as the experimental platform. It is configured with Intel Core i7 processor, 2.7GCPU dual-core 4G memory, and 500G hard drive. Use MATLAB7.0 and BP neural network toolbox as the experimental test environment.

The experimental data used in this paper come from the KDD CUP 99 test data set provided by Lincoln Laboratories. The detection data set contains a total of 4 types of attacks denial of service (DoS), R2L, scanning and probing (Probing), and U2R. The remaining data sets are all normal data. Since the data set has 41 characteristic attributes and a label attribute that distinguishes normal abnormal data, it contains continuous and discrete data and character strings, including 34-bit numeric attributes and 7-bit character attributes. The attack types in these data are not evenly distributed, and most of the attack types are DoS attacks. When probing and DoS attacks occur, their normal traffic and attack traffic are equal in number. However, the probability of U2R and R2L attacks is relatively small, and the attack traffic is very small compared to normal traffic. This is also in line with the runtime situation of cloud computing, which fully and truly reflects the security status of the cloud computing system. It also reflects the distribution of characteristics of various types of attacks.

### 5.2. Evaluation Index

This article adopts training accuracy rate (AC), false accuracy (FA), false-positive rate (FPR), and Kappa coefficient as the evaluation criteria of the experimental effect as follows:

The accuracy rate represents the proportion of the data set in which the model correctly classifies the actual value of the sample:

(9) $$\begin{array}{c} \text{AC}=\frac{Q}{S}\times 100\%, \end{array}$$

where *Q* is the number of samples correctly classified and *S* is the total number of samples.

FA represents the percentage of false acceptances and is defined as follows:

(10) $$\begin{array}{c} \text{FA}=\frac{W}{Z}\times 100\%, \end{array}$$

where *W* represents the number of normal samples that were falsely reported as intrusions and *Z* represents the number of normal samples.

FPR represents the proportion of false positives among all the samples that are actually negative:

(11) $$\begin{array}{c} \mathrm{FPR=}\frac{\mathrm{FN}}{\mathrm{TP+FN}}\times 100\%, \end{array}$$

where TP is a positive sample correctly classified by the model and FN is a positive sample incorrectly classified by the model.

### 5.3. Hyperparameter Analysis

This paper analyzes the influence of various factors on the detection effect from three aspects:

#### 5.3.1. The Impact of Input Dimensions on Detection Performance

Different input dimensions will affect the performance of the experiment. In order to find the appropriate input dimensions, this article sets 9 different sets of values to observe its influence on the experimental effect. Set the input dimension to 10–330 and the step size to 40. The experimental results are shown in Figure 7.

It can be seen from Figure 7 that when the input dimension is 10–330, AC shows an upward trend. When the input dimension is 250, the AC is the highest, and the difference between AC when the input dimension is 90 is small. When the input dimension is 250–330, the accuracy rate shows a downward trend. In terms of FA, when the input dimension is 290–330, FA shows a downward trend. When the input dimension is 210, its FA is the lowest, which is 17.78%. When the input dimension is 90–170, FA shows an upward trend. Considering experimental AC and FA comprehensively, when the dimension is 90, AC is higher and FA is lower. When the dimension is 240, AC is the highest but FA is also high. Therefore, the input dimension of the data in this paper is set to 90.

#### 5.3.2. The Effect of Convolution Kernel Size on Detection Performance

The size of the convolution kernel will directly affect the quality of feature extraction. The improper size of the convolution kernel will lead to incomplete feature extraction. In order to study the influence of the size of the convolution kernel on the detection performance, this paper sets up 9 convolution kernels of different sizes, 1–9, respectively. The experimental results are shown in Figure 8.

It can be seen from Figure 8 that the size of the convolution kernel has a significant impact on the accuracy. When the size of the convolution kernel is 4, the accuracy is the highest. The convolution kernel continues to increase, but its accuracy drops. Therefore, the convolution kernel should not be too large. The size of the convolution kernel has a relatively small effect on the false alarm rate, and when the size of the convolution kernel is 4, the false alarm rate is the lowest. In summary, when the size of the convolution kernel is 4, the experimental results obtained are better.

#### 5.3.3. BiLSTM Layer Structure Optimization Effect Comparison

This paper attempts to replace the BiLSTM unit with GRU and RNN units. At the same time, adjust the bidirectional LSTM layer structure to achieve a better classification effect. The model optimization effect comparison is shown in Table 1.

It can be seen from Table 1 that the RNN and GRU unit structure is relatively simple, and the training time required to build the model is relatively short. However, the accuracy rate is lower than that of the LSTM unit. Therefore, the following continues to optimize based on LSTM units. When the number of hidden layers of the LSTM layer is 2 and the number of hidden layer nodes is 20, the efficiency is improved without affecting the accuracy of the classifier. Therefore, this article will be further optimized based on the current structure.

### 5.4. Comparison of CNN-BiLSTM Feature Classification Performance of Different Classifiers

In order to illustrate the advantages of the features learned by CNN-BiLSTM combined with the performance of the C5.0 classifier, several machine learning classifiers such as KNN, J48, deep forest, naive Bayes, and random forest are selected for comparison experiments.  Table 2 shows the CNN-BiLSTM features of the NSL-KDD data set and the AC, FPR, and time (classifier construction and testing time) of several classifiers such as C5.0, KNN, and J48. It can be seen from Table 2 that the AC of the C5.0 classifier is 95.4%, the FPR is 5.4%, and the time is 8s. J48's classification AC is 59.2% and FPR is 44.8%, which is the lowest compared to other classifiers. The KNN classifier has a time of 32, which is the highest compared to several other classifiers. From the data in Table 2, it can be concluded that the performance of C5.0 classification of CNN-Bi LSTM features is the best.

### 5.5. Comparison with Other Detection Methods

This paper compares the CNN-BiLSTM method with methods based on AE-AlexNet [30] and SGM-CNN [31]. The comparison of the results of the three methods for four different attack types and AC, FA, and FPR under normal conditions is shown in Figures 9–11.

It can be seen from Figure 9 that the accuracy of the CNN-BiLSTM-based method is higher than that of the AE-AlexNet- and SGM-CNN-based methods because the LSTM method has the advantage of processing long-distance-dependent information. In this paper, the detection accuracy of the CNN-BiLSTM method for DoS, Normal, Probe, U2R, and R2L is 95.7%, 95.9%, 94.8%, 95.0%, and 96.1%, respectively. They are all higher than the other two methods, which proves the effectiveness of this method. The experimental results of the three methods in terms of FA are shown in Figure 10. It can be seen from Figure 10 that compared with the AE-AlexNet and SGM-CNN-based methods, the FA of the CNN-BiLSTM method in this paper is lower. The five types of FA for DoS, Normal, Probe, U2R and R2L are 4.1%, 4.0%, 3.2%, 4.7%, and 5.5%, respectively. The experimental results of the three methods in FPR are shown in Figure 11. It can be seen from Figure 11 that compared with the AE-AlexNet and SGM-CNN-based methods, the FPR of the CNN-BiLSTM method in this paper is lower. For the five types of DoS, Normal, Probe, U2R, and R2L, the FPRs are 7.5%, 6.9%, 6.2%, 6.4%, and 6.3%, respectively. The method in this paper uses CNN-BiLSTM to extract parallel local features of attribute information and extracts long-distance information-dependent features. Fully consider the influence between the attribute information before and after and introduce the attention mechanism and C5.0 decision tree to improve the classification accuracy of the method. Therefore, the detection effect is better.

## 6. Conclusion

This paper proposes a network intrusion detection method combining CNN-Bi LSTM and C5.0. First, the data extraction algorithm SamExtract is used to convert multiple traffic samples into grayscale images by performing operations such as data cleaning, data extraction, and data mapping on the original data set. Second, local parallel features are extracted through CNN to make up for the incomplete extraction of local features. And use bi-LSTM to extract long-distance-dependent features, so as to better consider the influence of the attributes before and after each attribute point in the sequence data, and reduce FA. Introduce attention mechanism to improve detection performance. Introduce the C5.0 decision tree to skip design feature selection and directly use the deep learning model to learn the representative features of high-dimensional data to better optimize the model. The experimental results show that the method proposed in this paper has higher AC and lower FA. However, the current network scale is expanding rapidly, and the types of traffic data are complex and large in scale.

In the follow-up work, the establishment of a network intrusion detection data set with a large amount of data, many new types of attacks, and a balanced sample is an important direction to improve the detection performance. In addition, it is necessary to simplify and improve the parameter adjustment process in the deep learning model training to improve the model time cost and detection effect.

## Figures and Tables

**Figure 1:** Schematic diagram of network intrusion detection system based on CNN.

**Figure 2:** Short- and long-term memory module.

**Figure 3:** Schematic diagram of boosting integration.

**Figure 4:** Schematic diagram of network intrusion detection based on CNN-BiLSTM.

**Figure 5:** CNN-BiLSTM model parameters.

**Figure 6:** Curve of acc-loss.

**Figure 7:** The influence of input latitude on AC and FA.

**Figure 8:** Impact of convolution kernel size on AC and FA.

**Figure 9:** Comparison of AC under different attack types.

**Figure 10:** Comparison of FA under different attack types.

**Figure 11:** Comparison of FPR under different attack types.

**Algorithm 1:** The pseudo code of the data extraction algorithm.

**Table 1:** Comparison of optimization effect of bi-LSTM layer structure.

Neuronal structure	Hidden units	Number of nodes	Iterations	Time (s)	Accuracy (%)
LSTM	1	10	60	1.462	94.22
LSTM	1	15	71	1.689	95.56
LSTM	1	20	80	1.921	95.32
LSTM	2	20	63	1.342	93.26
LSTM	3	20	92	1.253	93.87
GRU	1	20	66	1.452	94.22
RNN	1	20	55	1.997	95.76

**Table 2:** Comparison of BiLSTM feature classification performance of KDD CUP 99 data set.

Classifier	AC (%)	FPR (%)	Time (s)
KNN	78.1 (±0.0045)	23.4 (±0.0056)	32
J48	59.2 (±0.0055)	44.8 (±0.0155)	10
Deep forest	78.4 (±0.0100)	20.6 (±0.0010)	23
Naive Bayes	72.9 (±0.0050)	28.9 (±0.0150)	19
Random forest	85.2 (±0.0040)	15.2 (±0.0060)	28
The proposed method	95.4 (±0.0030)	5.4 (±0.0010)	8

## Data Availability

The data used to support the findings of this study are included within the article.
